# Identification of biomarkers and analysis of infiltrated immune cells in stable and ruptured abdominal aortic aneurysms

**DOI:** 10.3389/fcvm.2022.941185

**Published:** 2022-09-08

**Authors:** Yubin Chen, Tianyu Ouyang, Cheng Fang, Can-e Tang, Kaibo Lei, Longtan Jiang, Fanyan Luo

**Affiliations:** ^1^Department of Cardiac Surgery, Xiangya Hospital, Central South University, Changsha, China; ^2^Department of Endocrinology, Xiangya Hospital, Central South University, Changsha, China; ^3^The Institute of Medical Science Research, Xiangya Hospital, Central South University, Changsha, China; ^4^National Clinical Research Center for Geriatric Disorders, Xiangya Hospital, Central South University, Changsha, China

**Keywords:** abdominal aortic aneurysm, biomarker, aortic rupture, immune cells, macrophage, inflammation

## Abstract

**Objectives:**

The mortality rate of abdominal aortic aneurysm (AAA) is extremely high in the older population. This study aimed to identify potential biomarkers of AAA and aortic rupture and analyze infiltration of immune cells in stable and ruptured AAA samples.

**Methods:**

Raw data of GSE47472, GSE57691, and GSE98278 were downloaded. After data processing, the co-expression gene networks were constructed. Gene Ontology and pathway enrichment analysis of AAA- and aortic rupture-related gene modules were conducted using the Database for Annotation, Visualization, and Integrated Discovery. Gene set enrichment analysis (GSEA) and gene set variation analysis (GSVA) were used for further enrichment analysis. The CIBERSORT tool was used to analyze the relative abundance of immune cells in samples. Differentially expressed immune-related genes were analyzed between different samples. Predictive models were constructed *via* extreme gradient boosting, and hub genes were identified according to feature importance.

**Results:**

Blue and yellow modules were significantly related to AAA, and genes in these modules were associated with the aortic wall and immune response, respectively. In terms of aortic rupture, the most relevant module was significantly enriched in the inflammatory response. The results of GSEA and GSVA suggested that immune cells and the inflammatory response were involved in the development of AAA and aortic rupture. There were significant differences in the infiltration of immune cells and expression levels of immune-related genes among different samples. *NFKB1* might be an important transcription factor mediating the inflammatory response of AAA and aortic rupture. After the construction of a predictive model, *CD19*, *SELL*, and *CCR7* were selected as hub genes for AAA whereas *OAS3*, *IFIT1*, and *IFI44L* were identified as hub genes for aortic rupture.

**Conclusion:**

Weakening of the aortic wall and the immune response both contributed to the development of AAA, and the inflammatory response was closely associated with aortic rupture. The infiltration of immune cells was significantly different between different samples. *NFKB1* might be an important transcription factor in AAA and aortic rupture. *CD19*, *SELL*, and *CCR7* had potential diagnostic value for AAA. *OAS3*, *IFIT1*, and *IFI44L* might be predictive factors for aortic rupture.

## Introduction

Abdominal aortic aneurysm (AAA) is characterized by the weakening and dilatation of the abdominal aorta, which affects the infrarenal part most significantly (1). The diagnostic criterion of AAA is a maximum infrarenal abdominal aortic diameter of ≥ 30 mm (1), although there are other definitions of AAA in which its meaning is based on normalizing the aortic diameter to the body surface area (1, 2). Crucial risk factors for AAA include old age; male sex; smoking; a family history of AAA; the presence of other cardiovascular diseases (e.g., ischemic heart disease or peripheral artery disease), hypertension, and dyslipidemia (3, 4). According to recent ultrasonography-based screening studies, the prevalence of AAA in men > 65 years of age was 1–2% and that in women > 70 years of age was 0.5% (5–8). Aortic rupture is an important complication of AAA, which leads to 150,000–200,000 deaths each year worldwide, thus representing a severe threat to the older population (9, 10).

The predominant pathological changes in AAA are degeneration of the aortic media and apoptosis of vascular smooth muscle cells (VSMCs) (11). The extracellular matrix (ECM) is mainly synthesized and processed by VSMCs and plays an important role in the arterial function (12). Elastin and collagen are the main components of the ECM and can prevent the dilatation of the abdominal aorta and aortic rupture, respectively (13). Degradation of the ECM occurs largely due to an imbalance between amounts of active matrix metalloproteinases (MMPs) and their inhibitors (14). The inflammatory environment, reactive oxygen species (ROS), and endoplasmic reticulum stress can lead to the loss of VSMCs in AAA, which exacerbates the degradation of the ECM (15, 16). Infiltration of immune cells, including neutrophils, dendritic cells, macrophages, mast cells, B-cells, and T-cells, also contributes to the onset and development of AAA (17). However, the exact role of these immune cells in AAA remains unknown.

Ultrasonography and computerized tomography imaging are the most commonly used methods to diagnose AAA (1), but it is hard to diagnose AAA in the early stage because many patients with AAA are asymptomatic (18). In addition, the accuracy of predicting aortic rupture only based on the AAA diameter is low (19). Thus, further exploration of the mechanism of AAA formation and aortic rupture should be conducted to identify the potential biomarkers for AAA formation and aortic rupture, which may facilitate the early diagnosis of AAA and the prediction of aortic rupture. This study aimed to construct the AAA- and aortic rupture-related gene co-expression networks, analyze the infiltration of immune cells in AAA, identify differentially expressed inflammation-related genes (IRGs), and confirm the biomarkers involved in these processes using bioinformatics.

## Materials and methods

### Data acquisition and processing

The analysis process of this study is shown in Figure 1. The non-normalized data of GSE47472 (including eight normal abdominal aorta samples and 14 AAA samples), GSE57691 (including 10 normal abdominal aorta samples and 49 AAA samples), and GSE98278 (including 31 stable AAA samples and 17 ruptured AAA samples) were downloaded from the Gene Expression Omnibus (GEO) database^1^. All of these datasets were based on the same platform, GPL10558 (Illumina HumanHT-12 V4.0 expression BeadChip). The raw data of these datasets were normalized using the “Lumi” package in R software (version 4.1.2; R Foundation for Statistical Computing, Vienna, Austria) and the normalization process, including background correction, log2 transformation, and quantile normalization. Then, the data were annotated using the “dplyr” and “limma” packages in R software (version 4.1.2). The batch effect between each dataset was removed using the “sva” package in R software (version 4.1.2) and the data were then merged for further analysis; briefly, 94 AAA samples and 18 normal abdominal aorta samples were extracted from these datasets as merged dataset 1 to explore the potential mechanisms underlying AAA formation, whereas 94 stable AAA samples and 17 AAA rupture samples were obtained from these datasets as merged dataset 2 to identify rupture-related gene modules.

**FIGURE 1:** Flow chart diagram for analysis process in this study. WGCNA, weighted gene correlation network analysis; PPI, protein–protein interaction; GSEA, gene set enrichment analysis; GSVA, gene set variation analysis.

### Gene co-expression network construction by weighted gene correlation network analysis

Gene co-expression networks were constructed using the weighted gene correlation network analysis (WGCNA) package in R software (version 4.1.2) (20, 21). Soft-thresholding power was used to construct a weighted adjacency matrix. Relationships between a single gene and others in the analysis were incorporated, and the adjacency matrix was transformed into the topological matrix (TOM). Then, a hierarchical clustering analysis of genes was performed using 1 - TOM as the distance measure. Thereafter, modules were detected using a dynamic tree cut algorithm with a minimum module size of 50 and a minimum cut height of 0.99. The correlation between each module and the appearance of AAA or aortic rupture was calculated and shown in a heatmap. Finally, the most relevant gene modules were selected for further analysis.

### Gene ontology and Kyoto encyclopedia of genes and genomes pathway enrichment analysis of genes in the relevant gene modules

In this research, the Database for Annotation, Visualization, and Integrated Discovery (DAVID, 2021 Update^2^) was used to conduct gene ontology (GO) and Kyoto encyclopedia of genes and genomes (KEGG) pathways enrichment analysis of genes in the relevant gene modules.

### Construction of protein–protein interaction network and identification of candidate hub genes

Protein–protein interaction networks were constructed using the Search Tool for the Retrieval of Interacting Genes (STRING) online tool^3^ and visualized using Cytoscape software (version 3.9.1; Institute for Systems Biology, Seattle, WA, United States). Then, cytoHubba, a plugin of Cytoscape software was used to identify the top 10 genes *via* the MCC method, which were then regarded as candidate hub genes, and the corresponding protein–protein interaction (PPI) networks were constructed.

### Gene set enrichment analysis and gene set variation analysis

The gene set files used in this study were downloaded from the Molecular Signatures Database version 7.5.1^4^. The enrichment scores of GO and KEGG pathways terms in each group were calculated using the gene set enrichment analysis (GSEA) software (version 4.2.3) (22), and terms enriched in the AAA or aortic rupture group were identified. A nominal *p-*value of < 0.05 and false-discovery rate *q* value of < 0.25 were considered as significantly enriched in the AAA or aortic rupture group.

Gene set variation analysis was applied to evaluate GO and KEGG pathway terms enriched in each sample by converting the gene expression matrix into a gene set expression matrix using the GSVA package in R (version 4.1.2). After that, the differentially enriched terms between two groups were identified using R (version 4.1.2) with the threshold of *p* < 0.05. The differentially enriched terms were visualized using the “pheatmap” package in R (version 4.1.2).

### Analysis of infiltrated immune cells in samples

CIBERSORT^5^ is an algorithm that can analyze the relative abundance of 22 types of immune cells in each sample, including T-cells, B-cells, and macrophages (21). The parameters applied in this study were as follows: (I) 100 deconvolutions (Perm) and (II) *p* < 0.05. The analysis was conducted in R (version 4.1.2).

### Analysis of differentially expressed immune and inflammation-related genes and prediction of transcription factors

The IRG list was downloaded from Immport^6^. The differentially expressed IRGs (DEIRGs) between two groups were identified using R (version 4.1.2) with the threshold of *p* < 0.05. DAVID was used to identify the transcription factors (TFs) that could mediate these genes. The interaction between genes and TFs was visualized using Cytoscape (version 3.9.1).

### Preparation of the testing set

GSE7084 was selected as the testing set for the AAA predictive model and AAA-related hub genes, which included seven normal abdominal aorta samples and six AAA samples. Raw data were normalized following download from the GEO database using the “limma” package in R (version 4.1.2). Then, the data were annotated using the “dplyr” and “limma” package in R (version 4.1.2).

### Construction of a predictive model and identification of hub genes by extreme gradient boosting (XGBoost) analysis

To construct the AAA predictive model, all samples in merged dataset 1 were regarded as the training set and candidate hub genes of the AAA-related yellow module were selected as features. After the construction of a predictive model, GSE7084 was used as the testing set. To construct a rupture predictive model, samples in merged dataset 2 were divided into a training set (70%) and a testing set (30%) randomly and candidate hub genes of the rupture-related yellow module were selected as features. The rupture predictive model based on the training set was further validated in the testing set. The predictive models were constructed using the “xgboost” package in R (version 4.1.2), and hub genes were identified according to the rank of feature importance.

### Statistical analysis

The difference in relative expression levels of mRNA between different groups was analyzed with Student’s *t*-test. The proportion of each immune cell and the ratio of M1/M2 macrophages between different groups was analyzed by the Mann–Whitney *U* test. Pearson’s correlation analysis was used to analyze the relationship between inflammation genes and the infiltration of immune cells. A value of *p* < 0.05 was considered to be statistically significant. Statistical analyses were performed using SPSS version 19 (IBM Corporation, Armonk, NY, United States).

## Results

### Construction of abdominal aortic aneurysm- and aortic rupture-related gene co-expression networks

Soft threshold 12 was selected for AAA-related module construction. After analysis, 12 modules were obtained (Figure 2A); then, the relationship between different modules and AAA was analyzed and is shown in Figure 2B. The results indicated that the blue and yellow modules were significantly correlated with the appearance of AAA (blue module, *r* = –0.3, *p* = 0.001; yellow module, *r* = 0.27, *p* = 0.004). Therefore, the blue module and the yellow module were chosen for further analysis.

**FIGURE 2:** Construction of AAA- and aortic rupture-related gene co-expression networks using WGCNA and PPI networks of candidate hub genes. **(A)** Dendrogram and clustering for identification of gene co-expression modules of AAA-related merged dataset 1. **(B)** Correlation analysis of gene co-expression modules with AAA. The numbers above brackets were correlation coefficients and the numbers in brackets were *p*-values. **(C)** Dendrogram and clustering for identification of gene co-expression modules of aortic rupture-related merged dataset 2. **(D)** Correlation analysis of gene co-expression modules with aortic rupture. The numbers above brackets were correlation coefficients and the numbers in brackets were *p*-values. **(E,F)** The PPI networks of candidate hub genes of AAA-related blue module and yellow module, respectively. **(G)** The PPI networks of candidate hub genes of aortic rupture-related yellow module. AAA, abdominal aortic aneurysm; WGCNA, weighted gene correlation network analysis; PPI, protein–protein interaction.

Soft threshold 6 was selected for aortic rupture-related module construction and 17 modules were obtained (Figure 2E). Then, the correlation between different modules and aortic rupture was calculated, and the results suggested that the yellow module was the most relevant module (*r* = 0.46, *p* = 5e-07) (Figure 2F). Thus, the yellow module was selected for further analysis.

### Identification of candidate hub genes using protein–protein interaction network

The PPI networks of the AAA-related blue module, AAA-related yellow module, and aortic rupture-related yellow module were constructed *via* STRING and visualized using Cytoscape. The score of every node was calculated using the cytoHubba plugin for Cytoscape with the MCC method. Then, the top 10 nodes of each module were selected as candidate hub genes and are shown in Figures 2C,D,G.

### Gene ontology and Kyoto encyclopedia of genes and genomes pathway enrichment analysis of genes in the relevant gene modules

The enrichment analysis of the AAA-related blue module showed that the top 3 terms in the GO biological process (BP) subdivision were muscle contraction, cell adhesion, and angiogenesis, whereas the top three terms among the KEGG pathways were focal adhesion, ECM–receptor interaction, and hypertrophic cardiomyopathy (Table 1). The results of AAA-related yellow module suggested that the top three terms in GO BP included the immune response, T-cell activation, and the adaptive immune response and the top three terms in KEGG pathways included hematopoietic cell lineage, primary immunodeficiency, and the T-cell receptor signaling pathway (Table 1).

**TABLE 1:** Enrichment analysis of AAA and rupture-related gene modules.

Term	*P*-value	Benjamini
AAA-related blue module GO-BP		
Muscle contraction	5.987E-15	1.304E-11
Cell adhesion	3.207E-06	0.003
Angiogenesis	1.232E-05	0.009
Cell migration	2.111E-05	0.011
Actin filament organization	4.424E-05	0.019
AAA-related blue module KEGG pathway		
Focal adhesion	3.724E-06	0.001
ECM-receptor interaction	7.952E-05	0.001
Hypertrophic cardiomyopathy	9.489E-05	0.006
Vascular smooth muscle contraction	9.857E-05	0.006
Regulation of actin cytoskeleton	0.001	0.0232
AAA-related yellow module GO-BP		
Immune response	5.844E-12	7.778E-09
T-cell activation	4.800E-11	3.194E-08
Adaptive immune response	7.456E-08	3.308E-05
Regulation of immune response	1.687E-07	5.612E-05
T-cell costimulation	8.193E-07	<0.001
AAA-related yellow module KEGG pathway		
Hematopoietic cell lineage	1.748E-12	3.269E-10
Primary immunodeficiency	4.820E-07	4.507E-05
T-cell receptor signaling pathway	7.728E-06	<0.001
B cell receptor signaling pathway	9.066E-05	0.004
Cell adhesion molecules	<0.001	0.004
Rupture-related yellow module GO-BP		
Inflammatory response	3.032E-09	6.289E-06
Response to lipopolysaccharide	6.356E-07	<0.001
Angiogenesis	2.713E-05	0.008
Cellular response to interleukin-1	5.948E-05	0.0154
Positive regulation of p38MAPK cascade	<0.001	0.0221
Rupture-related yellow module KEGG pathway		
TNF signaling pathway	1.236E-07	3.064E-05
AGE-RAGE signaling pathway in diabetic complications	2.065E-06	<0.001
IL-17 signaling pathway	8.284E-06	0.001
HIF-1 signaling pathway	3.083E-05	0.002
Cytokine–cytokine receptor interaction	<0.001	0.005

AAA, abdominal aortic aneurysm; GO, Gene Ontology; BP, biological process; KEGG, Kyoto Encyclopedia of Genes and Genomes; ECM, extracellular matrix; MAPK, mitogen-activated protein kinase; TNF, tumor necrosis factor; AGE-RAGE, advanced glycation end-products receptor for advanced glycation end-products; IL-17, interleukin-17; HIF-1, hypoxia-induced factor-1.

The enrichment analysis of the aortic rupture-related yellow module indicated that the top 3 terms in the GO BP subdivision were inflammatory response, response to lipopolysaccharides, and angiogenesis, whereas the top three terms among the KEGG pathways were the tumor necrosis factor (TNF) signaling pathway, advanced glycation end-products receptor for advanced glycation end-products signaling pathway in diabetic complications, and interleukin (IL)-17 signaling pathway (Table 1).

### Gene set enrichment analysis and gene set variation analysis

Gene set enrichment analysis was conducted to understand the pathways enriched in different groups. The enrichment results of GO BP subdivision and KEGG pathway analysis demonstrated that positive regulation of leukocyte cell–cell adhesion, positive regulation of cell–cell adhesion, the adaptive immune response, cytokine–cytokine receptor interaction, the chemokine signaling pathway, and the NOD-like receptor signaling pathway were significantly enriched in the AAA group (Figures 3A–F). In terms of aortic rupture, the enrichment analysis results indicated that the serotonin receptor signaling pathway, regulation of peptidyl serine phosphorylation of STAT protein, serine phosphorylation of STAT protein, the Hedgehog signaling pathway, the mammalian target of rapamycin (mTOR) signaling pathway, and the vascular endothelial growth factor (VEGF) signaling pathway were significantly enriched in the aortic rupture group (Figures 3G–L).

**FIGURE 3:** The results of GSEA. **(A–C)** The GO-BP terms significantly enriched in AAA group. **(D–F)** The KEGG pathways significantly enriched in AAA group. **(G–I)** The GO-BP terms significantly enriched in aortic rupture group. **(J–L)** The KEGG pathways significantly enriched in aortic rupture group. GSEA, gene set enrichment analysis; GO-BP, Gene Ontology-biological process; AAA, abdominal aortic aneurysm; KEGG, Kyoto Encyclopedia of Genes and Genomes.

To further evaluate the pathway variations between different samples, GSVA was applied, and the results suggested that, compared to the normal abdominal aorta group, regulation of lymphocyte chemotaxis, protein poly ADP-ribosylation, regulation of T-cell chemotaxis, and graft-versus-host disease were significantly upregulated in the AAA group (Figures 4A,B). Besides, compared to the stable AAA group, sulfur metabolism, β-alanine metabolism, and valine leucine and isoleucine degradation were significantly increased in the ruptured AAA group (Figure 4C).

**FIGURE 4:** The results of GSVA. **(A)** Heatmap of top 20 significantly different GO-BP terms between normal abdominal aorta group and AAA group. **(B)** Heatmap of top 20 significantly different KEGG pathways between normal abdominal aorta group and AAA group. **(C)** Heatmap of significantly different KEGG pathways between stable AAA group and aortic rupture group. GSVA, gene set variation analysis; GO-BP, Gene Ontology-biological process; AAA, abdominal aortic aneurysm; KEGG, Kyoto Encyclopedia of Genes and Genomes.

### Changes in infiltrated immune cells in different samples

The overall relative abundances of 22 types of immune cells among the normal abdominal aorta samples and AAA samples are shown in Figure 5A. Then, the difference in the relative abundance of each type of immune cell between different groups was analyzed, and the results indicated that the proportions of activated memory CD4 T-cells and T follicular helper cells were significantly higher in the AAA group, whereas the proportion of M2 macrophages was significantly decreased in the AAA group (Figure 5B). We further compared the M1/M2 macrophage ratio and found that the ratio was significantly higher in the AAA group (Figure 5C).

**FIGURE 5:** Infiltration of immune cells in different samples. **(A)** Proportion of 22 kinds of immune cells in samples of AAA-related merged dataset 1. **(B)** The difference of infiltration of immune cells between normal abdominal aorta group and AAA group. The numbers in red represented *p*-value < 0.05. **(C)** The macrophage M1/macrophage M2 ratio in normal abdominal aorta group and AAA group. **(D)** Proportion of 22 kinds of immune cells in samples of aortic rupture-related merged dataset 2. **(E)** The difference of infiltration of immune cells between stable AAA group and aortic rupture group. The numbers in red represented *p*-value < 0.05. **(F)** The macrophage M1/macrophage M2 ratio in stable AAA group and aortic rupture group. AAA, abdominal aortic aneurysm. ***p < 0.001.

The relative abundances of 22 types of immune cells among the stable AAA samples and ruptured AAA samples are displayed in Figure 5D. Compared to the stable AAA group, the proportions of naïve CD4 T-cells, resting memory CD4 T-cells, activated memory CD4 T-cells, and activated dendritic cells were significantly greater in the ruptured AAA group, whereas the proportions of regulatory T-cells and M0, M1, and M2 macrophages, respectively, were significantly lower in the ruptured AAA group (Figure 5E). Further analysis indicated that the M1/M2 macrophage ratio was significantly higher in the ruptured AAA group (Figure 5F).

### Changes in inflammation-related genes in different groups and the relationship between inflammation-related genes and infiltration of immune cells

The DEIRGs between normal abdominal aorta samples and AAA samples were analyzed and the results revealed 453 DEIRGs, including 284 upregulated genes and 169 downregulated genes, with *p* < 0.05 (Figure 6A). Then, the TFs that could mediate these DEIRGs were predicted using DAVID. *STAT1*, *NFKB1*, *CREL*, and *P300* were the most relevant TFs considering the aforementioned DEIRGs, and the expression level of *NFKB1* was significantly upregulated in the AAA group (Figures 6B,C). The relationship among the top three upregulated DEIRGs, *NFKB1*, and significantly changed immune cells is displayed in Figure 6D. Similarly, we found 307 DEIRGs between the stable AAA group and ruptured AAA group, including 141 upregulated genes and 166 downregulated genes, with *p* < 0.05 (Figure 7A). *NFKB1*, *AP1*, *STAT1*, *BACH2*, and *STAT3* were the most relevant TFs considering these DEIRGs, and the expression level of *NFKB1* was also significantly increased in the ruptured AAA group (Figures 7B,C). In addition, the relationship among the top three upregulated DEIRGs, *NFKB1*, and significantly changed immune cells is displayed in Figure 7D.

**FIGURE 6:** Differentially expressed immune and inflammation-related genes (DEIRGs) between normal abdominal aorta group and AAA group. **(A)** The volcano plot of DEIRGs between normal abdominal aorta group and AAA group. Dots in green: downregulated gene, dots in red: upregulated gene. **(B)** The PPI network of DEIRGs and upstream transcription factors. **(C)** The expression level of NFKB1 in normal abdominal aorta group and AAA group. **(D)** The relationship between top three upregulated DEIRGs, NFKB1, and significantly changed immune cells. Dots in blue: normal abdominal aorta samples, dots in red: AAA samples. AAA, abdominal aortic aneurysm; PPI, protein–protein interaction; NFKB1, nuclear factor kappa B 1; corr, correlation coefficient. *p < 0.05, **p < 0.01, ***p < 0.001.

**FIGURE 7:** Differentially expressed immune and inflammation-related genes (DEIRGs) between stable AAA group and aortic rupture group. **(A)** The volcano plot of DEIRGs between stable AAA group and aortic rupture group. Dots in green: downregulated gene, dots in red: upregulated gene. **(B)** The PPI network of DEIRGs and upstream transcription factors. **(C)** The expression level of NFKB1 in stable AAA group and aortic rupture group. **(D)** The relationship between top three upregulated DEIRGs, NFKB1, and significantly changed immune cells. Dots in blue: stable AAA samples, dots in red: aortic rupture samples. AAA, abdominal aortic aneurysm; PPI, protein–protein interaction; NFKB1, nuclear factor kappa B 1; corr, correlation coefficient. *p < 0.05, **p < 0.01, ***p < 0.001.

### Construction of the predictive model and identification of hub genes

The top 10 candidate hub genes in the AAA-related yellow module were selected as features to construct an AAA predictive model. The accuracy of this model was 0.7692 in testing set GSE7084 (Table 2). The identification of hub genes was performed according to the rank of feature importance, and *CD19*, *SELL*, and *CCR7* were the top three features (Figure 8A). The expression levels of *CD19*, *SELL*, and *CCR7* in the training set are shown in Figure 8B and were further validated in testing set GSE7084 (Figure 8C).

**TABLE 2:** The predictive ability of XGBoost model in GSE7084.

		XGBoost model predicted		Accuracy
		Normal	AAA	
Actual	Normal	5	1	0.7692
	AAA	2	5	

XGBoost, extreme gradient boosting; AAA, abdominal aortic aneurysm.

**FIGURE 8:** Identification of hub genes. **(A)** The rank of feature importance in AAA predictive model. **(B)** The expression levels of CD19, SELL, and CCR7 in AAA-related merged dataset 1. **(C)** The expression levels of CD19, SELL, and CCR7 in testing set GSE7084. **(D)** The rank of feature importance in aortic rupture predictive model. **(E)** The expression levels of OAS3, IFIT1, and IFI44L in aortic rupture-related merged dataset 2. AAA, abdominal aortic aneurysm. *p < 0.05, **p < 0.01, ***p < 0.001.

The construction of an aortic rupture predictive model was based on the top 10 candidate hub genes in the aortic rupture-related yellow module. During the construction process, four features were excluded because they did not contribute to the model (Figure 8D). The accuracy of this model was 0.9697 in the testing set (Table 3). The top three features were *OAS3*, *IFIT1*, and *IFI44L* (Figure 8D), and the expression levels of these genes are demonstrated in Figure 8E.

**TABLE 3:** The predictive ability of XGBoost model in the testing set.

		XGBoost model predicted		Accuracy
		Stable	Rupture	
Actual	Stable	26	0	0.9697
	Rupture	1	6	

XGBoost, extreme gradient boosting.

## Discussion

The prevalence of AAA is derived from ultrasonography screening programs of a few developed countries. According to these ultrasonography screening programs, the prevalence of AAA is approximately 1–2% in men > 65 years of age and 0.5% in women > 70 years of age (5–8). The exact prevalence of AAA in developing countries is unclear due to the lack of ultrasonography screening programs but has increased over the past two decades according to the literature (5, 17). Generally, smoking, older age, positive family history, male sex, hypertension, and dyslipidemia are significantly associated with the appearance of AAA (23–25). It was reported that the incidence of AAA increases by 6% per decade in men after the age of 65 years (26). In the developed countries, AAA-related death has been the 12–15th leading cause of death in those > 55 years of age, and aortic rupture is a predominant cause of AAA-related death (12, 27). The main treatment for AAA is surgical procedures such as endovascular aortic repair (EVAR) and open repair surgery (17). Currently, there is no drug-based therapy able to inhibit the AAA growth or aortic rupture (18, 28, 29). Therefore, further exploration of the mechanisms of AAA formation or aortic rupture is needed to identify new therapeutic targets or biomarkers that may allow for diagnosis and cure in early stages or the prediction of aortic rupture.

GSE47472, GSE57691, and GSE98278 were chosen and selectively merged for further bioinformatics analysis. These three datasets were detected using the same platform, which facilitates the consistency of the detection process. Considering the bioinformatics studies of Xie et al. (30) and Yuan et al. (31), this study contained more datasets and samples than either of the former. Moreover, instead of identifying differentially expressed genes directly, AAA- and aortic rupture-related gene co-expression networks were constructed using WGCNA first in this research. After evaluating the correlation between AAA-related gene modules and the appearance of AAA, the results revealed that the absolute correlation coefficient of the blue module was the largest among these modules, with *p* < 0.05. However, we also noticed that the absolute correlation coefficient of the yellow module was close to that of the blue module, so the blue and yellow modules were both selected for further analysis. The results of enrichment analysis of the AAA-related blue module indicated that genes in this module were involved in processes, including muscle contraction, structural constituent of muscle, and vascular smooth muscle contraction, both of which are closely related to the aortic wall. This finding is consistent with current opinions about the development of AAA. One of the main causes of AAA is a progressive degenerated abdominal artery wall, which is characterized by degradation of the ECM in the adventitia and the loss of VSMCs (32). The main components of the ECM are microfibrillar (elastin and collagen) and microfibrillar (fibronectin and fibrillin) structures of crosslinked proteins, which maintain the function of the artery wall and resist its dilatation and rupture (13). Increases in serine proteases and activated MMPs lead to degradation of the ECM and eventually result in dilation and rupture of the abdominal artery wall (33, 34). VSMCs synthesize ECM components and secret enzymes such as lysyl oxidase, thus involving themselves in the maturation of fibrillar structures in the ECM (12). The proteolytic, inflammatory, and oxidative environments in the abdominal artery wall could lead to the detachment and death of VSMCs and affect the synthesis of ECM components (15, 35).

Genes in the AAA-related yellow module were significantly enriched in terms like immune response, T-cell activation, and the B-cell receptor signaling pathway. Similarly, the results of GSEA and GSVA suggested that positive regulation of leukocyte cell–cell adhesion, the chemokine signaling pathway, and regulation of lymphocyte chemotaxis were significantly enriched in the AAA group. These results indicate that the immune and inflammation response is another important mechanism of AAA. Previous studies have revealed that both innate and adaptive immunity contribute to the development of AAA (12). In healthy individuals, the media of the abdominal aorta is an immune-privileged site devoid of capillaries, while the adventitia of the abdominal aorta is fully vascularized with many capillaries, enabling immune cell diapedesis and triggering an immune response (36). Under the AAA condition, the relative hypoxia environment in the abdominal aorta would induce the expression of VEGF in macrophages and VSMCs and eventually lead to angiogenesis in the adventitia and media of the abdominal aorta (37). The innate immune activity includes diapedesis, activation, and death of polymorphonuclear leukocytes in AAA, whereas leukocytes release proteases, oxidant peptides, myeloperoxidase, and pro-inflammatory factors, both of which could accelerate the development of AAA (32). However, the proteolytic and/or oxidative environments in the abdominal artery wall of patients with AAA can trigger an adaptive immune response, which commonly takes place in the adventitia of the abdominal artery (36). The adaptive immune response in AAA is associated with the formation of an adventitial tertiary lymphoid organ (TLO), whose center is composed of B-cells and surrounded by endothelial venules, follicular dendritic cells, and T follicular helper cells. The function of the TLO includes antibody production and immunoglobulin switching (38). Our bioinformatics analysis further confirmed that the immune and inflammation response is a key process in the development of AAA.

Aortic rupture is the main cause of death in patients with AAA, so it is necessary to further explore the potential mechanisms underlying aortic rupture. The enrichment analysis of the aortic rupture-related yellow module revealed that genes in this module were associated with the cytokine-mediated signaling pathway and inflammatory response. In addition, the results of GSEA indicated that the STAT, mTOR, and VEGF signaling pathways were significantly enriched in the aortic rupture group. The traditional risk factors for aortic rupture include AAA size, wall thickness, hypertension, smoking, advanced age, and systemic inflammation (39). There is an increasing number of studies suggesting that inflammation is significantly associated with aortic rupture. Aurelian et al. reported that the neutrophil-to-lymphocyte ratio (NLR) was increased in patients with aortic rupture compared to patients with intact AAAs, and an NLR of > 5 indicated a fivefold increased risk of aortic rupture (40). Studies by Treska et al., Cheuk et al., and Wallinder et al. demonstrated that pro-inflammatory cytokines such as IL-6, IL-8, and TNF-α were upregulated in the plasma and aneurysm tissue of patients with AAA rupture (41–43). STAT signaling pathways could mediate cellular activity, including the inflammatory response, and Wang et al. reported that the STAT4 signaling pathway is involved in the development and rupture of AAA (44). There are also studies demonstrating that the mTOR and VEGF signaling pathways play the important roles in the development of AAA (45, 46), but their roles in aortic rupture remain unclear.

According to the results of enrichment analysis, GSEA, and GSVA, immune and inflammatory responses participate in the development of AAA and aortic rupture. Thus, we further investigated the infiltration of immune cells in each sample using CIBERSORT. The results showed that the proportion of M2 macrophages was significantly decreased in AAA samples compared to normal abdominal artery samples and the M1/M2 macrophage ratio was significantly greater in AAA samples compared to normal abdominal artery samples. Studies have demonstrated that M1 is a pro-inflammatory phenotype of macrophages, whereas M2 is an anti-inflammatory phenotype of macrophages (47). Our findings further validated the idea that the aneurysmal wall is under a severe inflammatory condition. In addition, macrophages secret VEGF and MMPs, which could provoke angiogenesis in the adventitia and media of the abdominal aorta and result in weakening of the aneurysmal wall (37). The results also indicated that the proportions of activated memory CD4 T-cells and T follicular helper cells were significantly higher in AAA samples. Pathological study has confirmed the infiltration of T-cells in the aneurysmal wall (48). Galle et al. reported that CD4 + T-cells infiltrated into the aneurysmal wall exhibit a unique activated memory phenotype and could produce interferon-γ at a high level (49). Gao et al. also showed that infiltration of activated memory CD4 T-cells and T follicular helper cells was significantly increased in AAA samples using CIBERSORT (50). However, there remain few studies documenting the exact role of T-cells in AAA, which requires further investigation. Thus, we compared the infiltration of immune cells in stable AAA samples and ruptured AAA samples. Surprisingly, the proportions of M0, M1, and M2 macrophages, respectively, were all significantly lower in ruptured AAA samples than stable AAA samples, but the M1/M2 macrophage ratio was still significantly higher in the ruptured AAA samples, revealing their severe inflammatory environment. In contrast to our findings, a bioinformatics analysis performed by Lei et al. suggested that the proportions of M0, M1, and M2 macrophages were similar among stable AAA samples and ruptured AAA samples (51). This difference in results might be due to the choice of dataset selected for analysis. In this research, GSE47472, GSE57691, and GSE98278 were selected to investigate the potential mechanism of aortic rupture, whereas Lei et al. (51) only chose GSE98278 for further analysis. In addition, we found that the proportions of naïve CD4 T-cells, resting memory CD4 T-cells, and activated memory CD4 T-cells were significantly lower in stable AAA samples compared to ruptured AAA samples. These findings were consistent with those of Amin et al., whose research indicated that the reduced infiltration of CD4 + T-cells could attenuate inflammation, preserve integrity of the artery, and reduce the risk of aortic rupture (52). We also noticed that the proportion of regulatory T-cells was significantly lower in ruptured AAA samples. Similarly, Ait-Oufella et al. found that natural regulatory T-cells limit angiotensin II-induced AAA formation and rupture in mice (53).

We continued to investigate the DEIRGs between different samples. There were 453 DEIRGs between normal abdominal aorta samples and AAA samples, and *STAT1*, *NFKB1*, *CREL*, and *P300* were the most relevant TFs that could mediate these DEIRGs according to the enrichment analysis of DAVID. Among these TFs, NFKB1 was significantly increased in AAA samples. Similarly, there were 307 DEIRGs between stable and ruptured AAA samples; *NFKB1*, *AP1*, *STAT1*, *BACH2*, and *STAT3* were the most relevant TFs, and *NFKB1* was significantly upregulated in ruptured AAA samples. Studies have demonstrated the importance of the NFKB1 signaling pathway in the development of AAA (54, 55), suggesting that the NFKB1 signaling pathway might be a promising therapeutic target of AAA.

As mentioned above, most patients with AAA are asymptomatic in the early stage and it is hard to predict aortic rupture in these individuals (18). Therefore, in a subsequent study, we investigated which potential biomarkers had diagnostic value for AAA or could predict aortic rupture. First of all, we constructed an AAA predictive model using XGBoost, which could effectively avoid the overfitting problem (56). The candidate hub genes of the AAA-related yellow module were selected as features of this model. These genes were inflammation-related and their expression levels can also change in peripheral blood, which allows us to conveniently detect them with limited damage. The accuracy of the AAA predictive model in testing set GSE7084 was 0.7692. Thereafter, genes were ranked according to feature importance, and the top three genes were *CD19*, *SELL*, and *CCR7*, which were selected as hub genes. CD19 is a marker of B-cells and the micro-array study of Biros et al. indicated that CD19 was significantly increased in AAA samples (57). Shi et al. found that CD19-positive cells were significantly infiltrated in AAA samples using immunohistochemical staining (58). Marie et al. reported that SELL was associated with the development of AAA (59). Furthermore, several bioinformatics studies revealed that *CCR7* is one of the hub genes of AAA (60, 61). Our findings and previous investigations suggest that these genes might be involved in the development of AAA and could be potential biomarkers for AAA, but their diagnostic value needs further validation.

An aortic rupture predictive model was constructed using XGBoost and the candidate hub genes of the aortic rupture-related yellow module were features in the model. The accuracy of this model in the inner testing set was 0.9697 and the top 3 hub genes were *OAS3*, *IFIT1*, and *IFI44L*. OAS3 is a member of the 2’-5’-oligoadenylate synthetase family and is involved in immune responses, which could restrict the replication of certain types of viruses (62, 63). Interferon-induced protein with tetratricopeptide repeats (IFIT) 1 is a member of the IFIT family and plays an important role in antiviral processes, and research has revealed that IFIT1 is involved in the development of systemic lupus erythematosus (SLE) (64, 65). Interferon-induced protein 44-like is an interferon-induced gene overexpressed in patients with SLE that might be a drug target of SLE (66). However, the relationships between these three genes and aortic rupture are unclear, and the predictive values of aortic rupture require further exploration.

The main limitation of these hub genes is that they are not suitable for clinical diagnosis because they were detected in AAA tissue samples. However, these genes were found to be closely related to the immune or inflammation process, and expression levels of these genes might change in peripheral blood. Further research needs to be done to investigate the changes of these genes in peripheral blood. Other genes that could interact with these hub genes should be investigated as well. On the other hand, non-coding RNAs, including microRNAs, circular RNAs, and long non-coding RNAs, could be promising biomarkers for some diseases (67). In the next step, a competing endogenous RNA network of these hub genes should be constructed and the RNAs with diagnostic value identified.

In conclusion, weakening of the artery wall and the immune response significantly contributed to the development of AAA, and the inflammatory response was one of the most important factors leading to aortic rupture. The infiltration of immune cells was significantly different between normal abdominal artery samples and AAA samples, stable AAA samples, and ruptured AAA samples. NFKB1 might be an important TF that mediates the inflammatory response of AAA and aortic rupture. CD19, SELL, and CCR7 had potential diagnostic value for AAA. OAS3, IFIT1, and IFI44L may be predictive factors for aortic rupture.

## Data availability statement

Publicly available datasets were analyzed in this study. This data can be found here: https://www.ncbi.nlm.nih.gov/geo/query/acc.cgi?acc=GSE47472, https://www.ncbi.nlm.nih.gov/geo/query/acc.cgi?acc=GSE57691, https://www.ncbi.nlm.nih.gov/geo/query/acc.cgi?acc=GSE98278, and https://www.ncbi.nlm.nih.gov/geo/query/acc.cgi?acc=GSE7084.

## Author contributions

YBC analyzed the data, completed the figures, and wrote the manuscript. TYOY and CF processed the raw data. C-eT, KBL, LTJ, and FYL designed the research. LTJ and FYL reviewed and edited the manuscript. All authors contributed to the article and approved the submitted version.

## Footnotes

1
https://www.ncbi.nlm.nih.gov/gds

2
https://david.ncifcrf.gov/home.jsp

3
https://cn.string-db.org/

4
http://www.gsea-msigdb.org/gsea/msigdb/index.jsp

5
https://cibersort.stanford.edu/

6
https://www.immport.org/home
